The article "Gene expression profiles analysis identifies key genes for acute lung injury in patients with sepsis" was retracted in 2015. Reasons: misconduct by a third party; compromised peer review.

# Gene expression profiles analysis identifies key genes for acute lung injury in patients with sepsis

**DOI:** 10.1186/s13000-014-0176-x

**Published:** 2014-09-26

**Authors:** Zhiqiang Guo, Chuncheng Zhao, Zheng Wang

**Affiliations:** Department of Thoracic surgery, Putuo Hospital,Shanghai University of Traditional Chinese Medicine, No. 164 Lan Xi Road, Shanghai, 200062 China

**Keywords:** Acute lung injury, Differentially expressed genes, Functional enrichment analysis, Gene regulatory network

## Abstract

**Background:**

To identify critical genes and biological pathways in acute lung injury (ALI), a comparative analysis of gene expression profiles of patients with ALI + sepsis compared with patients with sepsis alone were performed with bioinformatic tools.

**Methods:**

GSE10474 was downloaded from Gene Expression Omnibus, including a collective of 13 whole blood samples with ALI + sepsis and 21 whole blood samples with sepsis alone. After pre-treatment with robust multichip averaging (RMA) method, differential analysis was conducted using simpleaffy package based upon t-test and fold change. Hierarchical clustering was also performed using function hclust from package stats. Beisides, functional enrichment analysis was conducted using iGepros. Moreover, the gene regulatory network was constructed with information from Kyoto Encyclopedia of Genes and Genomes (KEGG) and then visualized by Cytoscape.

**Results:**

A total of 128 differentially expressed genes (DEGs) were identified, including 47 up- and 81 down-regulated genes. The significantly enriched functions included negative regulation of cell proliferation, regulation of response to stimulus and cellular component morphogenesis. A total of 27 DEGs were significantly enriched in 16 KEGG pathways, such as protein digestion and absorption, fatty acid metabolism, amoebiasis, etc. Furthermore, the regulatory network of these 27 DEGs was constructed, which involved several key genes, including protein tyrosine kinase 2 (PTK2), v-src avian sarcoma (SRC) and Caveolin 2 (CAV2).

**Conclusion:**

PTK2, SRC and CAV2 may be potential markers for diagnosis and treatment of ALI.

**Virtual Slides:**

The virtual slide(s) for this article can be found here: http://www.diagnosticpathology.diagnomx.eu/vs/5865162912987143

## Background

Acute lung injury (ALI), also called acute respiratory distress syndrome (ARDS), is a systemic inflammatory response syndrome characterized by refractory hypoxemia and respiratory distress [1]. It can be caused by all kinds of pathogenic factors inside and outside the lungs (such as serious infection, aspiration, sepsis, trauma and shock), principally sepsis [1-3]. ALI appears the earliest and is with the highest incidence in patients with sepsis [4,5]. Although advancements in critical care has improved the survival among patients with ALI, the mortality is still as high as 40% and the rate of survivors with significant pulmonary impairment is approximately 50% [6].

The major challenge is accurate and early diagnosis of patients with ALI. The current clinical criteria include pulmonary edema, hypoxemia and widespread capillary leakage. However, there’s a discrepancy between clinical criteria and histological autopsy findings [7]. Intraobserver variability in diagnosis is also unavoidable. Thus, the difficulties in diagnosis make it necessary to identify biomarkers for ALI. Many studies have been carried out in different sample sources like pulmonary edema [8], fluid blood and urine [9,10]. In addition, gene expression profiles analysis has been conducted, microarray technology enables a global investigation of gene expression and promotes identification of biomarkers of potential diagnostic and prognostic significance [11-13]. Moreover, it provides insights on the molecular mechanisms underlying the ALI [14,15].

In 2009, Howrylak *et al.* used a gene expression microarray data to develop a gene signature of ARDS/ALI between patients with ALI + sepsis and patients with sepsis alone, and obtained an eight-gene expression profile that can distinguish patients with ALI + sepsis from patients with sepsis alone accurately [11]. In 2013, Chen *et al.* downloaded the expression profile deposited by Howrylak *et al.* [11], and identified the differentially expressed genes (DEGs) between patients with ALI + sepsis and patients with sepsis alone and obtained 12 DEGs. They also constructed protein-protein interaction network (PPI) and conducted functional enrichment analysis, and obtained two networks (OCLN and HLA-DQB1), as well as enriched 7 significant functions in OCLN network and 5 functions in HLA-DQB1 network [16]. Using the same data by Howrylak *et al*. [11], we aimed to further screen the DEGs. Especially, hierarchical clustering of genes and samples by the expression level of the DEGs was performed. And the potential functions of the DEGs were analyzed by Gene Ontology (GO) and pathway enrichment analyses. In addition, the interaction relationships between these DEGs significantly enriched in Kyoto Encyclopedia of Genes and Genomes (KEGG) pathways were investigated by regulatory network.

## Methods

### Gene expression data

Expression profile of GSE10474 [11] was downloaded from Gene Expression Omnibus database (GEO, http://www.ncbi.nlm.nih.gov/geo/), including 13 whole blood samples with ALI plus sepsis (ALI + sepsis) and 21 whole blood samples with sepsis alone. Patients admitted to the Medical Intensive Care Unit (MICU) of the University of Pittsburgh Medical Center for no more than 48 h who received mechanical ventilation were regarded suitable for the study. And appropriate patients were recruited from the MICU between February 2005 and June 2007. Gene expression was measured using Affymetrix Human Genome U133A 2.0 Array (Affymetrix Inc., Santa Clara, California, USA).

### Pre-treatment and differential analysis

Raw data were read with package affy of *R* [17] in Bioconductor [18]. Background correction, normalization and calculation of expression value were performed using the robust multichip averaging (RMA) method. Differential analysis was conducted using package Simpleaffy [19] based upon t-test and fold change. The adjusted p-value < 0.05 and |log_2_fold-change (FC)| > 1 were set as the cut-off criteria.

### Clustering analysis

As a widely used data analysis tool, hierarchical clustering is aimed to build a binary tree of the data that successively combines similar point groups, and visualization of the tree offers a useful summary of this data [20]. Hierarchical clustering of genes and samples by the expression level of the DEGs was performed using hierarchical cluster function hclust from base package stats of *R* [17].

### Functional enrichment analysis

To obtain an in-depth analysis of the DEGs from the functional levels, biological process (BP), cell components (CC) and molecular function (MF) functional enrichment analysis was conducted using iGepros [21] (http://www.biosino.org/iGepros/index.jsp). P-value < 0.05 was set as the cut-off to screen out significant GO terms and KEGG pathways. Significant KEGG pathways were visualized using KEGG Mapper tools [22].

### Gene regulatory network construction

A total of 27 DEGs were significantly enriched in 16 KEGG pathways. In addition, regulators of these DEGs and various regulatory relationships (such as activation, inhibition, phosphorylation, compound binding, coexpression, and protein-protein interaction) were retrieved from the 16 KEGG pathways. The gene regulatory network was visualized by Cytoscape [23]. Proteins in the network served as the 'nodes', and each pairwise protein interaction (referred to as edge) was represented by an undirected link. The property of the network was analyzed with the plug-in network analysis.

## Results

### Differentially expressed genes

According to the criteria (adjusted p-value < 0.05 and |log_2_FC| > 1), a total of 128 DEGs were identified in patients with ALI + sepsis compared with patients with sepsis alone, including 47 up-regulated genes and 81 down-regulated genes.

### Functional enrichment analysis results

Top 10 GO terms (BP, CC and MF) are shown in Table 1. Negative regulation of cell proliferation, regulation of response to stimulus and cellular component morphogenesis were included in the list.

**Table 1:** **Top 10 Gene Ontology (GO) terms enriched in the differentially expressed genes**

**Ontology**	**GO_ID**	**P-value**	**Count**	**Term**
BP	GO:0008285	7.85E-05	12	negative regulation of cell proliferation
	GO:0032502	0.000116652	47	developmental process
	GO:0060161	0.000160183	2	positive regulation of dopamine receptor signaling pathway
	GO:0040011	0.000192818	19	locomotion
	GO:0032989	0.000216136	16	cellular component morphogenesis
	GO:0048732	0.000225085	8	gland development
	GO:0007267	0.000237497	18	cell-cell signaling
	GO:0048583	0.000451816	27	regulation of response to stimulus
	GO:0000904	0.000507026	13	cell morphogenesis involved in differentiation
	GO:0018108	0.000561365	6	peptidyl-tyrosine phosphorylation
CC	GO:0005578	3.27E-05	11	proteinaceous extracellular matrix
	GO:0005576	7.15E-05	30	extracellular region
	GO:0005938	0.0007889	6	cell cortex
	GO:0005615	0.0011351	14	extracellular space
	GO:0044420	0.0013032	6	extracellular matrix part
	GO:0016323	0.0020977	7	basolateral plasma membrane
	GO:0005624	0.0052989	13	membrane fraction
	GO:0009986	0.005548	8	cell surface
	GO:0005901	0.0059176	3	caveola
	GO:0033593	0.0069353	1	BRCA2-MAGE-D1 complex
MF	GO:0019534	0.0004939	2	toxin transporter activity
	GO:0008504	0.0010276	2	monoamine transmembrane transporter activity
	GO:0042803	0.0019488	10	protein homodimerization activity
	GO:0030165	0.0023021	4	PDZ domain binding
	GO:0005515	0.0023215	55	protein binding
	GO:0005201	0.0026418	4	extracellular matrix structural constituent
	GO:0008144	0.0027622	4	drug binding
	GO:0022804	0.0029877	8	active transmembrane transporter activity
	GO:0015101	0.0037119	2	organic cation transmembrane transporter activity
	GO:0050750	0.0043105	2	low-density lipoprotein particle receptor binding

BP, biological process; CC, cellular component; MF, molecular function; Count, number of differentially expressed genes.

A total of 120 KEGG pathways were enriched for the 128 DEGs, including 16 significantly enriched pathways (Table 2), such as fatty acid metabolism, beta-alanine metabolism, ErbB signaling pathway, ECM-receptor interaction, protein digestion and absorption, bile secretion and gastric acid secretion.

**Table 2:** **Significant Kyoto Encyclopedia of Genes and Genomes (KEGG) pathways enriched in the differentially expressed genes**

**KEGG_ID**	**P-value**	**Count**	**Size**	**Term**
K04974	0.0058969	4	81	Protein digestion and absorption
K00071	0.0066462	3	43	Fatty acid metabolism
K05146	0.0149273	4	106	Amoebiasis
K00410	0.0164577	2	22	beta-Alanine metabolism
K04950	0.021009	2	25	Maturity onset diabetes of the young
K05100	0.0248666	3	70	Bacterial invasion of epithelial cells
K04976	0.0258013	3	71	Bile secretion
K04971	0.0287182	3	74	Gastric acid secretion
K05310	0.0296041	2	30	Asthma
K04514	0.0313484	4	133	Cell adhesion molecules (CAMs)
K04510	0.0333551	5	200	Focal adhesion
K00040	0.0333724	2	32	Pentose and glucuronate interconversions
K04512	0.0408489	3	85	ECM-receptor interaction
K04012	0.0432936	3	87	ErbB signaling pathway
K05330	0.0435527	2	37	Allograft rejection
K05215	0.0458106	3	89	Prostate cancer

### The regulatory network of the DEGs

A total of 27 DEGs were significantly enriched in 16 KEGG pathways. Regulators of these DEGs and various regulatory relationships (such as activation, inhibition, phosphorylation, compound binding, co-expression, and protein-protein interaction) were retrieved from the 16 KEGG pathways. The regulatory network was constructed (Figure 1). Especially, protein tyrosine kinase 2 (PTK2), v-src avian sarcoma (SRC), and Caveolin 2 (CAV2) may be hub genes for ALI. Furthermore, in the regulatory network of the DEGs, SRC had interaction relationships with PTK2, as well as CAV2 were targeted by SRC.

**Figure 1:** **The regulatory network of the differentially expressed gene.** The protein products of the DEGs are in red. The size of a node correlates with the number of interactions of the node while the thickness of an edge correlates with the edge betweenness of the edge.

## Discussion

A total of 128 DEGs were identified in sepsis-induced ALI compared with sepsis, including 47 up-regulated genes and 81 down-regulated genes. Functional enrichment analysis indicated that several metabolism-related KEGG pathways were enriched in the DEGs, including fatty acid metabolism and beta-alanine metabolism. Several signaling pathways were also significantly enriched in the DEGs, such as ECM-receptor interaction and ErbB signaling pathway. Especially, the regulatory network of the 27 DEGs involved several key genes (such as PTK2, SRC and CAV2).

PTK2 and SRC both were implicated in cell growth and they were down-regulated in ALI [24,25]. Since repair of damaged endothelium is important in recovery from ALI and increased circulating endothelial progenitor cells are associated with survival [26], we speculated that modulation of these cell growth-related genes could provide another way to treat the disease. Besides, digestion-related pathways were also disclosed in the DEGs, such as protein digestion and absorption, bile secretion and gastric acid secretion, which might be explained by poor health of patients with ALI.

As an important family for intracellular signal transduction, Src protein tyrosine kinases (PTKs) are associated with acute inflammatory responses [27-30]. It’s not expression level alteration of Src PTK but its activation may be related to reperfusion-induced lung injury [31]. As inhibitor of SRC activation, PP2 can attenuate alveolar macrophage priming for improved lipopolysaccharide responsiveness and induce a modest reduction in lung injury [31-33]. And chemical inhibitors directly or indirectly regulating Src PTKs have been used as potential drugs for the treatment of lung injury [34]. In the regulatory network of the DEGs, SRC had interaction relationships with PTK2. These declared that SRC might play a role in ALI by mediating PTK2.

Correspondingly, negative regulation of cell proliferation was the most significant biological pathways in GO enrichment analysis. CAV2 is a major component of the inner surface of caveolae. It is involved in essential cellular functions, including signal transduction, lipid metabolism, cellular growth control and apoptosis. Its related family member CAV1 is reported to be a critical regulator of lung injury [35]. De Almeida *et al.* find that genetic ablation of caveolin-2 sensitizes mice to bleomycin-induced injury [36]. We speculated that CAV2 might play a role in the pathogenesis of ALI. In the regulatory network of the DEGs, CAV2 were targeted by SRC, indicating that CAV2 might also be involved in ALI by mediating SRC.

To further look into the molecular mechanisms underlying ALI, a gene regulatory network was constructed for the DEGs and various regulatory relationships were visualized. PTK2, SRC and CAV2 are hub genes in the network. As discussed above, these genes are related to cell proliferation. The gene regulatory network further demonstrated the close association between cell growth and ALI.

## Conclusion

Overall, we carried out an integrated bioinformatics analysis of genes which may play a role in ALI. A total of 128 DEGs were identified, including 47 up-regulated genes and 81 down-regulated genes. Functional enrichment analysis showed that cell proliferation and lipid metabolism were closely related to ALI. Moreover, relevant genes like PTK2, SRC and CAV2 might be potential biomarkers for diagnosis and treatment of ALI.
